The article "Meta-Analysis of the Diagnostic Value of Tracer Staining Technology Based on Nanocarbon Suspension in Sentinel Lymph Node Biopsy of Breast Cancer" was published in 2022. Journal: Comput Math Methods Med.

# Meta-Analysis of the Diagnostic Value of Tracer Staining Technology Based on Nanocarbon Suspension in Sentinel Lymph Node Biopsy of Breast Cancer

**DOI:** 10.1155/2022/2299852

**Published:** 2022-05-12

**Authors:** Luhua Xia, Le Chong, Zinan Lu, Xinhua Wang, Zhanfei Dong, Yanping Zhao, Cheng Chang, Gang Sun

**Affiliations:** ^1^Department of Nuclear Medicine, The Affiliated Cancer Hospital of Xinjiang Medical University, Urumqi, Xinjiang 830011, China; ^2^Department of Ultrasonography, The Affiliated Cancer Hospital of Xinjiang Medical University, Urumqi, Xinjiang 830011, China; ^3^Department of Radiotherapy, The Affiliated Cancer Hospital of Xinjiang Medical University, Urumqi, Xinjiang 830011, China; ^4^Department of Breast and Thyroid Surgery, The Affiliated Cancer Hospital of Xinjiang Medical University, Xinjiang Cancer Center/Key Laboratory of Oncology of Xinjiang Uyghur Autonomous Region, Urumqi, Xinjiang 830011, China

## Abstract

**Objective:**

To evaluate the diagnostic value of the nanometer carbon suspension tracer staining technique in sentinel lymph node biopsy of breast cancer is the objective of this study.

**Methods:**

The PubMed, Embase, Cochrane Library (Central), and Web of Science (SCI Expanded), and Chinese databases (CNKI, VIP, Wan Fang, and CBM) were systematically searched for studies on the diagnostic value of nanocarbon suspension in sentinel lymph node biopsy of breast cancer. Two reviewers independently assessed the methodological quality of each study using the QUADAS-2 tool. The extracted valid data were calculated using Meta-Disc1.4 software and tested for heterogeneity. STATA14.0 software was selected for sensitivity analysis of the included studies, and publication bias was assessed using Deeks' forest plot asymmetry test.

**Results:**

A total of 10 studies were obtained. The pooled data were as follows: sensitivity, 0.92 (0.88~0.95); specificity, 0.99 (0.98~1.00); positive likelihood ratio, 69.24 (30.34~158.02); negative likelihood ratio, 0.09 (0.06~0.13); and the combined diagnostic odds ratio, 747.40 (285.77~1954.76), AUC = 0.9881. Nanocarbon suspension tracers have an accuracy rate of 98.81% in the diagnosis of sentinel lymph nodes in breast cancer.

**Conclusion:**

Tracer staining technology based on nanocarbon suspension can accurately assess the status of lymph nodes in sentinel lymph node biopsy of breast cancer and has good stability and operability, which is worthy of clinical promotion.

## 1. Introduction

Breast cancer is an important cause of human suffering and premature death in women worldwide [1]. The lymphatic system is the most common vehicle of metastasis in breast cancer, in which sentinel lymph nodes (SLNs) are the first locations for primary tumor spread [2]. Clinically, systemic metastasis is often judged according to the results of pathological examination. Understanding the status of sentinel lymph nodes in breast cancer is an important basis for us to evaluate axillary lymph node metastasis. The traditional axillary lymph node dissection (ALND), large-scale clearance of axillary lymph nodes on the affected side, is associated with larger incision, deeper operation location, and higher operation cost. And after the operation, it is easy to have upper limb lymph node edema, and patients have large scars, which bring more pain to the patients. SLN biopsy (SLNB) only removes SLNs for pathological confirmation of metastasis, and whether to expand the scope of operation is determined by the pathological results. If there is no metastasis of sentinel lymph nodes, we will not consider expanding the scope of incision.

The article "Meta-Analysis of the Diagnostic Value of Tracer Staining Technology Based on Nanocarbon Suspension in Sentinel Lymph Node Biopsy of Breast Cancer" was published in 2022. Journal: Comput Math Methods Med.

SLNB was introduced in the early 1990s as a less invasive procedure than complete lymph node dissection and can be used for histopathological evaluation of SLNs in place of axillary lymph node dissection (ALND) for staging in patients with early breast cancer. SLNB is the first choice to evaluate the axillary staging of breast cancer patients. This method can accurately predict the status of the axillary lymph nodes and avoid axillary lymph node dissection for SLN-negative breast cancer patients. Additionally, SLNB can prevent surgical trauma and upper limb lymph node edema, reduce the cost of surgery, and improve the quality of life in patients postoperatively, and it can also retain a certain number of axillary lymph nodes so that it can continue to maintain the immune barrier against tumor [3–5]. Safe and efficient methods to improve the detection rate and accuracy of SLNs have been the focus of research in recent years.

The traditional tracer methods of SLNB include dye method, radionuclide tracer method, and dye combined radionuclide method, but they all have some shortcomings. Some new tracer methods are produced continuously, such as nanocarbon suspension (NCS) tracer method, contrast-enhanced ultrasound tracer method, indocyanine green fluorescence method, and superparamagnetic iron oxide tracer method [6–10].

The dye method is easy to operate and easy to obtain. The most commonly used dye is methylene blue, which has low molecular weight, strong binding to tissue protein, and simple operation. It can be injected around the areola 10-30 minutes before operation without special equipment and low price. It is the most widely used tracer at present. The reported complications include allergic reaction, local inflammation, skin and fat necrosis, and skin staining. By radionuclide tracer method, the detection rate of SLN is high, and the false-negative rate is low. The configured 99mTc was injected subcutaneously around the areola 6 hours before operation, and the hot spot signal area identified by the gamma detector during the operation was SLN. Because the radionuclide tracer needs to be injected before operation, the patient has obvious pain during injection, the operation process is complex, the price is high, and the corresponding instruments and equipment are needed in clinical application, and the cooperation of nuclear medicine department is needed, so it is difficult to carry out in grassroots hospitals. Dye method combined with radionuclide method has high SLN detection rate and low false-negative rate, but the operation process is complex, and it also needs the cooperation of professional instruments and equipment and nuclear medicine, which is high in cost and difficult to popularize. Ultrasound tracer is a safe, economical, and noninvasive technique, which can dynamically observe the lymphatic drainage channel and imaging lymph nodes in real time and can identify SLN. According to the contrast-enhanced mode of SLN, we can judge whether SLN has metastasis or not, but the disadvantage is that there is a certain false-negative rate. Indocyanine green fluorescence method and real-time lymphatic system imaging can help the chief surgeon to choose the surgical incision, thus reducing the difficulty of operation, simple operation, safe nonradiation, and high detection rate of SLN. However, due to the attenuation of fluorescence by subcutaneous tissue, its application in obese patients with BMI>30 is limited, the research time is still short, and there is no recognized technical standard at present. The superparamagnetic iron oxide nanoparticle tracer method is simple, safe, and noninvasive, and the detection rate of sentinel lymph nodes is similar to that of radionuclides, but it has the problem of false negative and needs further study.

The article "Meta-Analysis of the Diagnostic Value of Tracer Staining Technology Based on Nanocarbon Suspension in Sentinel Lymph Node Biopsy of Breast Cancer" was published in 2022. Journal: Comput Math Methods Med.

NCS is the first new type of third-generation specific lymph node tracer approved by the State Food and Drug Administration (SFDA) [11]. Patented preparation technology is used to grind activated carbon particles into 21-nm particles, and then polyvinylpyrrolidone (PVP) and normal saline are added to prepare the NCS, which makes it possible to be widely used in surgery for thyroid cancer, gastric cancer, cervical cancer, colorectal cancer, and others. It has also been used as a lymph node tracker and has achieved good results [12–20].

A meta-analysis was conducted to systematically evaluate the diagnostic value of NCS in SLNB of breast cancer.

## 2. Materials and Methods

The meta-analysis is based on the Preferred Reporting Items for Systematic Review and Meta-Analysis (PRISMA) [21]. We included a study of patients with breast cancer confirmed by pathology. During sentinel lymph node biopsy, NCS was used as a tracer to identify lymph nodes. Histopathological results were used to compare and report true-positive (TP), false-positive (FP), true-negative (TN), and false-negative (FN) results. The type of nanocarbon study was a diagnostic test.

### 2.1. Study Search Strategy

PubMed, Embase, Cochrane Library (Central), and Web of Science (SCI Expanded), and Chinese databases (CNKI, VIP, Wan Fang, and CBM) were searched by computer for relevant research up to January 2022. Subject words plus free words were used for retrieval using the following terms with no language restrictions:

Step 1: (Carbon nanoparticle suspension; Nano-carbon; Nano carbon; Nanogate Carbon; Carbon Nanoparticles; Nano carbon suspension; NCS) connect with OR: “Carbon nanoparticle suspension” OR “Nano-carbon” OR “Nano carbon” OR “Nanogate Carbon” OR “Carbon Nanoparticles” OR “Nano carbon suspension” OR “NCS”.

Step 2: (Breast Neoplasms; Breast tumor; Mammary cancer; Breast carcinoma; Breast Cancer), connect with OR: “Breast Neoplasms” OR “Breast Carcinoma” OR “Breast tumor” OR “Mammary cancer” OR “Breast carcinoma” OR “Breast Cancer”.

Step 3: (Sentinel Lymph Node; Lymph Node, Sentinel; Lymph Nodes, Sentinel; Sentinel Lymph Nodes; Sentinal Node; Node, Sentinal; Nodes Sentinal; Sentinal Nodes) connect with OR: “Sentinel Lymph Node” OR “Lymph Node, Sentinel” OR “Lymph Nodes” OR “Sentinel Lymph Nodes” OR “Sentinal Node” OR “Node, Sentinal” OR “Nodes Sentinal” OR “Sentinal Nodes”.

Step 4: The above three are searched by AND connection in the following manner: (“Carbon nanoparticle suspension” OR “Nanocarbon” OR “Nanocarbon” OR “Nanogate Carbon” OR “Carbon Nanoparticles” OR “Nanocarbon suspension” OR “NCS”) AND (“Breast Neoplasms” OR “Breast tumor” OR “Mammary cancer” OR “Breast carcinoma” OR “Breast Cancer”) AND (“Sentinel Lymph Node” OR “Lymph Node, Sentinel” OR “Lymph Nodes” OR “Sentinel Lymph Nodes” OR “Sentinal Node” OR “Node, Sentinal” OR “Nodes Sentinal” OR “Sentinal Nodes”). The list of qualified studies was also screened to find other related articles. The search strategy for relevant Chinese publications was similar to that for English publications.

### 2.2. Study Selection

The inclusion criteria were as follows: (1) studies on the application of sentinel lymph node biopsy in breast cancer using NCS; (2) only studies enrolling females; (3) cases of breast cancer confirmed by pathological biopsy; (4) negative results of preoperative physical examination of axillary lymph nodes; (5) no previous history of axillary surgery or breast radiotherapy; (6) women with breast cancer who were not pregnant or lactating; and (7) complete 2 × 2 table data.

The article "Meta-Analysis of the Diagnostic Value of Tracer Staining Technology Based on Nanocarbon Suspension in Sentinel Lymph Node Biopsy of Breast Cancer" was published in 2022. Journal: Comput Math Methods Med.

The exclusion criteria were as follows: (1) duplicate studies; (2) case reports, reviews, letters, comments, and systematic evaluation studies; (3) experiments involving animals; and (4) incomplete 2 × 2 table data.

### 2.3. Data Extraction

Two investigators independently used predesigned forms to extract relevant data. Any differences were discussed until consensus was reached. The following information was extracted from each study: serial number, name of the first author, year of publication, age range of the patient, preoperative stage of the patient, and true-positive, false-positive, true-negative, and false-negative results.

### 2.4. Quality Assessment

A total of 10 studies were included, and the method quality was independently assessed by two authors responsible for data extraction using the Diagnostic Accuracy Research Quality Assessment (QUADAS2) [22]. If the two readers disagreed, a third reader became involved, and the final result was determined by consensus. No authors were involved in the 10 included studies. The QUADAS-2 checklist consists of four areas: patient selection, indicator testing, reference criteria, and process/scheduling. Based on several questions, a bias risk assessment was conducted for each of the four areas. The software used was Review Manager 5.4 (Cochrane Collaboration Group).

### 2.5. Statistical Analysis

The present meta-analysis was conducted by using Meta DiSc1.4 (XI Cochrane Colloquium, Barcelona, Spain) and Stata14.0 (Stata Corporation, College Station, TX, USA) software. Sensitivity (SEN), specificity (SPE), 95% confidence interval(CI), positive likelihood ratio (+ LR), negative likelihood ratio(-LR), and diagnostic odds ratio (DOR) were extracted or calculated from the study and then used to evaluate the accuracy of the diagnosis. The receiver working characteristic (SROC) summary curve was constructed, the area under the curve (AUC) was calculated, and the diagnostic accuracy was analyzed. Stata software version 14.0 was used to determine the heterogeneity between studies; the inconsistency index (*I*^2^) was calculated based on the *Q* statistics of the chi-square test (25-50%, 51-75%, >75%; low, medium, and high heterogeneity, respectively). An *I*^2^ value greater than 50% was considered to indicate significant heterogeneity [23]. The *I*^2^ from a random effects model was less than that of a fixed-effects model [24].

## 3. Results

### 3.1. Literature Search

The flowchart of literature retrieval is shown in Figure 1. According to the retrieval strategy, a total of 402 articles were initially retrieved, including 215 duplicate studies; 23 reviews, reports, and systematic reviews; and 7 animal experiments. A total of 165 studies were eliminated after reading the corresponding abstract because the content failed to meet the requirements of this study. For the same reason, 8 studies were eliminated after carefully reading the full text, and 2 studies were eliminated due to incomplete data. Finally, 10 studies were included in this study. No additional literature met the requirements of this study (Figure 1).

The article "Meta-Analysis of the Diagnostic Value of Tracer Staining Technology Based on Nanocarbon Suspension in Sentinel Lymph Node Biopsy of Breast Cancer" was published in 2022. Journal: Comput Math Methods Med.

### 3.2. Study Characteristics

The detailed characteristics of the studies are listed in Table 1. Ten studies (882 patients, all female, aged 24 to 83 years) were conducted in China from 2011 to 2018; 9 studies were written in Chinese, and 1 study was written in English. Because NCS is a third-generation specific tracer approved by the China Food and Drug Administration, it is only sold in China and has not entered the international market; therefore, there is no relevant research in other countries (Table 1).

### 3.3. Quality Assessment

The QUADAS2 quality evaluation tool was used to evaluate the literature quality, and the results showed that all the included studies were of relatively high quality. In terms of the reference standard, none of the 10 studies addressed whether the interpretation of the gold standard strictly complies with the principle of blind law; thus, there is a high concern about the reference standard. However, there were no concerns about the choice of patients and index testing. Ten studies have qualified to be included in the meta-analysis based on QUADAS-2 assessments (Figure 2).

### 3.4. Exploration of Heterogeneity

Threshold effect heterogeneity: The data were imported into Meta DiSc1.4 soft for analysis, and the Spearman correlation coefficient between the sensitivity logarithm and (1-specificity) logarithm was -0.274, which was not significant. By drawing a symmetrical SROC curve, there was no “shoulder arm shape,” suggesting that there was no heterogeneity caused by the threshold effect in this study.

Nonthreshold effect heterogeneity: The Cochran *Q* test of the DOR was 2.27, *P* = 0.9865 > 0.001, suggesting that there was no heterogeneity caused by the nonthreshold effect in this study.

The Galbraith diagram drawn using Stata software version 14.0 (Stata Corporation, College Station, TX, USA) shows that all studies are on both sides of the red effect line and within the green confidence interval, suggesting that there is no heterogeneity in this study (Figure 3).

The article "Meta-Analysis of the Diagnostic Value of Tracer Staining Technology Based on Nanocarbon Suspension in Sentinel Lymph Node Biopsy of Breast Cancer" was published in 2022. Journal: Comput Math Methods Med.

### 3.5. Meta-Analysis

The figure clearly shows the sensitivity (*I*^2^ = 0) and specificity (*I*^2^ = 4.9%). Using the fixed-effects model, the combined sensitivity was 0.92 (0.88-0.95), the combined specificity was 0.99 (0.98-1.00), and the combined positive likelihood ratio was 69.24 (30.34-158.02). The likelihood ratio of negative merger was 0.09 (0.06-0.13) (Figure 4). The odds ratio of combined diagnosis was 747.40 (285.77-1954.76), and the AUC was 0.9881.

### 3.6. SROC Curve Drawing

Drawing the AUC = 0.9881 based on the SROC curve using NCS as a tracer, the diagnostic accuracy in SLNB of breast cancer was as high as 98.81%, and the diagnostic accuracy was high (Figure 5).

### 3.7. Sensitivity Analysis Test

Stata software version 14.0 (Stata Corporation, College Station, TX, USA) was used for sensitivity analysis of the data in this study. From the following figure, we can clearly see that there is strong sensitivity of the original study (No. 8). The other nine original studies did not cause the results to be sensitive, and the results of this study are relatively stable (Figure 6).

### 3.8. Publication Bias

Using Stata software version 14.0, Deeks' funnel plot asymmetry test was selected to test the publication bias of the data. The chart shows that the scatter asymmetry is distributed on both sides of the regression line, and the funnel diagram is asymmetrical; publication bias was evident at *P* < 0.001 (Figure 7).

### 3.9. Clinical Utility of NCS in SLNB

Figure 8 shows the likelihood nomograph used by Fagan NCS in SLNB. The prior probability is set to 20%. NCS is used as a tracer for SLNB of breast cancer. If the result is positive, the metastasis probability of pre-SLN is 99%. If the result is negative, the metastasis probability of SLN is 2%.

## 4. Discussion

A comprehensive analysis of 10 studies (882 patients) showed that the combined sensitivity, specificity, and positive likelihood ratio of NCS in SLNB of breast cancer were 0.92 (0.88-0.95), 0.99 (0.98-1.00), and 69.24 (30.34-158.02), respectively. The combined negative likelihood ratio was 0.090. The combined DOR was 747.40 (285.77-1954.76), AUC = 0.9881. The diagnostic accuracy of NCS as a tracer in sentinel lymph node biopsy of breast cancer is as high as 99.81%, suggesting that NCS is a desirable diagnostic tool in sentinel lymph node biopsy of breast cancer.

In 1994, Giuliano et al. [25] reported that blue staining was used to predict SLNB. In 1998, Krag et al. [26] first reported the application of radionuclide tracer in the prediction of breast cancer SLNB. Among the three traditional SLN tracer methods, dye method is simple, intuitive, practical, low-cost, and does not need professional equipment, but it is time-consuming and causes large damage. The advantages of nuclide method are clear preoperative positioning, strong surgical pertinence, and small damage, but the disadvantages are radioactive contamination, expensive equipment, and complex preparation process. The selection of good tracer is the key to the success of SLNB.

The article "Meta-Analysis of the Diagnostic Value of Tracer Staining Technology Based on Nanocarbon Suspension in Sentinel Lymph Node Biopsy of Breast Cancer" was published in 2022. Journal: Comput Math Methods Med.

Zhang, L et al. [27] considered that the value of NCS tracers in the identification and prediction of SLNB was satisfactory. Wu, X et al. [28] confirmed the feasibility and accuracy of carbon nanoparticles in the localization of SLNs in patients with breast cancer. Carbon nanoparticles are very useful in SLN detection in institutions where radioisotopes cannot be obtained. Many studies suggest that carbon nanosuspension can effectively detect the anatomical location and number of sentinel lymph nodes in thyroid cancer, gastric cancer, cervical cancer, colorectal cancer, and other tumors and improve the accuracy of SLN examination [12–20].

As a new type of tracer, the imaging principle of NCS is that the average diameter of NCS particles is 150 nm, which is larger than the diameter of capillaries (20-50 nm); therefore, the particles cannot enter capillaries, but they can smoothly pass through the lymphatic capillaries (diameter 120-500 nm). When NCS suspension is injected into the tissue around the tumor, macrophages phagocytose the charcoal particles and carry them into the lymphatic capillaries and lymph nodes, staining the lymph nodes black. As a result, because the hydrostatic pressure in the tissue space is greater than the pressure in the lymphatic capillaries, NCS will not enter the tissue space and stain the local tissue black. Compared with traditional dyes, the lymph nodes and lymphatics are clear with no diffusion to the surrounding tissue. Additionally, there are no obvious adverse reactions in clinical application. NCS is relatively inexpensive and does not require the use of special detection equipment during the operation. The safety of NCS location has been confirmed in animal experiments and human experiments [29, 30]. Its advantages are as follows: fast absorption by lymphoid tissue, long retention time in SLNs, ease of use, moderate price, and safe and nontoxic. Additionally, NCS will not cause background staining by water-soluble reagents such as methylene blue [31–33]. In all included studies, no allergic reactions, local inflammatory reactions, or skin and fat necrosis were reported; however, staining of the skin was common with NCS.

However, the use of NCS for sentinel lymph node biopsy also has some potential risks, in addition to the skin contamination problem, that is, the existence of false negative, which is an important reason affecting the promotion and application of SLNB. We believe that there may be the following reasons for false negative: (1) It is related to tumor staging. The large volume of tumor cells and a large number of axillary lymph node metastasis may be due to the tumor thrombus formed by tumor cells and the local tissue of the focus after compression. The blind end of the lymphatic vessels or some branches of lymphatic capillaries hinders the migration of phagocytes in the lymphatic capillaries, thus affecting the entry of NCS into the lymphatic system and preventing SLN from black staining. (2) It is related to the age of the tumor patients. The lymphoid tissue may atrophy in older tumor patients. (3) It is related to the location of tumor. Tumors located in the outer upper quadrant are easy to oppress and block the lymphatic vessels, thus affecting the entry of NCS into the lymphatic system of the lateral group, so that SLN cannot be black-stained, resulting in false-negative cases. (4) It is related to the different injection points of tracers. Although subareolar injection is a rapid method to trace lymph nodes, there are some differences according to different types of lymphatic drainage at different injection sites.

The article "Meta-Analysis of the Diagnostic Value of Tracer Staining Technology Based on Nanocarbon Suspension in Sentinel Lymph Node Biopsy of Breast Cancer" was published in 2022. Journal: Comput Math Methods Med.

This study has the following limitations: (1) Although this study involved an extensive search, unpublished literature could not be obtained; therefore, potential publication bias cannot be ruled out. In-depth subgroup analysis can provide instructive information for diagnosis and identification. Due to the limited information provided by the original included studies, no further subgroup analysis was performed. The quality of the original literature may also affect the results of the meta-analysis. (2) Because NCS is a third-generation specific tracer approved by the China Food and Drug Administration, it is only sold in China and does not enter the international market. As a result, there is no relevant research in other countries, and no regional or ethnic studies are involved, which may have a certain impact on the results of the meta-analysis; (3) Most of the studies did not report the length of time before performing SLNB after injection. Additionally, it was necessary to further increase the sample size to analyze the difference in the injection time of NCS and to discuss whether the time difference after injection had any effect on the diagnosis of SLNs.

In summary, NCS makes up for many shortcomings of traditional tracers [33–39]. It has the advantages of small dosage, accurate location, strong staining specificity, and rapid development. Additionally, NCS, a moderate-cost tracer, is easy to use, safe and non-polluting, harmless to the human body, and shows long residence time in lymph nodes. Collectively it has a widely application prospect. This meta-analysis shows that the NCS tracer staining technique has high diagnostic accuracy in sentinel lymph node biopsy of breast cancer. Clinicians can select NCS for lymph node localization for breast cancer patients as an alternative to other methods and associated problems such as methylene blue staining time and many complications, making CNS worthy of clinical application and promotion.

The article "Meta-Analysis of the Diagnostic Value of Tracer Staining Technology Based on Nanocarbon Suspension in Sentinel Lymph Node Biopsy of Breast Cancer" was published in 2022. Journal: Comput Math Methods Med.

NSC remains in lymph nodes for a long time, and it is easy to use, moderate price, safe, and nontoxic. To improve the effectiveness of NSC application, it is necessary to (1) accelerate the promotion of NCS into the international market and make it play an important role in lymph node diagnosis. (2) The price of NCS is slightly higher than that of methylene blue injection, which is a commonly used staining tracer, and controlling its price is also an important aspect of popularization and application. (3) To clarify and promote the safety and importance of the application of nanomedicine in biomedicine, with the deepening of the application and research of new nanomaterials and nanotechnology in the medical field, more and more nanodrug preparations are or have been put into clinical research and put on the market, which are full of opportunities and challenges in the future. The combination of nanotechnology and medicine has promoted the improvement of basic medical research technology, the innovation of clinical diagnosis technology, and the improvement of treatment level. It is believed that NCS will become an important lymph node tracer in the near future.

## Figures and Tables

**Figure 1:** The study selection process.

**Figure 2:** Methodological quality graph (a) and methodological quality summary (b).

**Figure 3:** Galbraith diagram.

**Figure 4:** The forest plot of NCS as a tracer in breast cancer SLNB sensitivity (a), specificity (b), positive likelihood ratio (c), and negative likelihood ratio (d).

**Figure 5:** The SROC curve.

**Figure 6:** The sensitivity analysis of the 10 included studies is shown, with study No. 8 displaying strong sensitivity (a). After removing the sensitivity analysis chart of study No. 8, the results of this study were stable (b).

**Figure 7:** Publish a bias test.

**Figure 8:** Probability of the Fagan likelihood nomograph and NCS in detecting lymph node metastasis by SLNB.

**Table 1:** Summary data of 10 included studies.

No.	First author	Time	Country	Age	Preoperative staging	TP	FP	FN	TN	Total
No. 1	Bo Yan	2011	China	28-69	T1-T2N0M0	52	0	8	92	152
No. 2	Wenbin Guo	2012	China	24-68	T1-T2 N0M0	14	0	1	19	34
No. 3	Zongyi Chen	2012	China	39-62	T1-T2 N0M0	22	0	2	20	44
No. 4	Dagong Song	2013	China	30-83	T1-T2 N0M0	28	0	2	60	90
No. 5	Tielei Tang	2013	China	60-81	T1-T2 N0M0	5	0	1	15	21
No. 6	Shuanggen Lei	2014	China	27-73	T1-T2 N0M0	20	0	1	35	56
No. 7	Haitao Guan	2015	China	26-67	T1-T2 N0M0	31	0	2	54	87
No. 8	Xinzheng Wang	2016	China	27-73	T1-T2 N0M0	14	5	1	229	249
No. 9	Ningbin Du	2016	China	22-68	T1-T2 N0M0	28	0	2	28	58
No. 10	Liulu Zhang	2018	China	25-77	T1-T3 N0M0	47	0	2	42	91

TP: true positive; FP: false positive; FN: false negative; TN: true negative.

The article "Meta-Analysis of the Diagnostic Value of Tracer Staining Technology Based on Nanocarbon Suspension in Sentinel Lymph Node Biopsy of Breast Cancer" was published in 2022. Journal: Comput Math Methods Med.

## Data Availability

The data used to support the findings of this study are available from the corresponding author upon request.

## Abbreviations

SLN: Sentinel lymph nodes
SLNB: Sentinel lymph node biopsy
ALND: Axillary lymph node dissection
NCS: Nanocarbon suspension
PLR: Positive likelihood ratio
SFDA: State Food and Drug Administration
NLR: Negative likelihood ratio
DOR: Diagnostic odds ratio.
